# New Pyroptosis -Associated Gene Signature for Overall Survival Forecast among Patients Suffering from Hepatocellular Carcinoma

This article has been retracted.

**DOI:** 10.1155/2022/6365485

**Published:** 2022-04-15

**Authors:** Cheng He, Ke You

**Affiliations:** ^1^Department of Hepatobiliary Surgery, Affiliated Hospital of Xiangnan University, Chenzhou 423000, China; ^2^Department of Hepatobiliary Surgery, The Second Affiliated Hospital of Chongqing Medical University, Chongqing 400010, China

## Abstract

Due to the heterogeneity of tumors, we do not understand the given effect of pyroptosis on hepatocellular carcinoma (HCC) fully, particularly its influences on prognosis. The paper aims at exploring the prognostic value of pyroptosis-associated genes and its role in immune status in HCC. A multigene prognostic signature is set up by utilizing the least absolute shrinkage and choosing operator Cox exploration. The comparison of survival between different risk groups is made with the Kaplan–Meier exploration and Cox regression. LASSO Cox regression analysis is adopted to set up a pyroptosis-associated gene signature (*CEP55* and *MMP1*). By comparing with the group at low risks, the high-risk group displayed greatly decreased OS. The fatidic ability of the prognostic gene signature is confirmed by the receiver-running feature curve analysis. According to multivariate Cox exploration, the risk mark is an independent predicting agent for OS. A new signature established with two pyroptosis-associated genes can be adopted for prognostic forecast and influence the immune situation in HCC.

## 1. Introduction

Hepatocellular carcinoma (HCC), a malignant tumor, is the fifth most frequent cancer and the second major cause of cancer-associated death across the world. HCC is mostly an issue of the less developed areas where approximately 83% (or 50% in China alone) of the 854,000 new cancer cases across the world happened in 2018. Being the second most frequent causes of cancer death, it is predicted that HCC oversees nearly 810,000 deaths in 2018 (8.2% of the total deaths of all cancers). Thus, liver cancer still shows very poor prognosis with a total proportion of mortality to incidence of 0.95 [1, 2]. In the past thirty years, the sobering outcome of patients with hepatocellular carcinoma has not been significantly enhanced because of high heterogeneity. Given the poor prognosis, especially for advanced HCC patients, the molecular mechanisms for the occurrence of HCC needs to be understood urgently.

As a programmed cell death adjusted by gasdermin, pyroptosis has characteristics such as continuously expanding cells until the fracture of cell membrane, resulting in releasing cell amount, and stimulating a great inflammatory response. As a significant natural immune response of the body, pyroptosis exerts an important effect on the fight against tumors. However, the effect of pyroptosis on the HCC growth and prognosis is still uncertain. In this research, we are trying to dig the correlation between pyroptosis and the appearance and growth of liver cancer, establish a prognostic model, and offer a novel idea for treating HCC.

The paper uses the data of two independent HCC cohorts: The Cancer Genome Atlas (TCGA) (https://portal.gdc.cancer.gov/repository) and the International Cancer Genomics Consortium (ICGC) (https://dcc.icgc.org/projects/LIRI-JP). Pyroptosis-associated genes (*n* = 52) are obtained from prior reviews [3–6]. TCGA cohort is used to explore the prognostic value of the associated genes for HCC. Genes with a *p*-value <0.05 validated by univariate Cox regression exploration are regarded prognostic-associated genes (PRGs) [7–12]. Next, the PRGs are in accordance with cluster exploration by the R package “Consensus Cluster Plus.” The overall survival (OS) diversity between various subtypes is analyzed with the Kaplan–Meier approach. The chi-square test is adopted for comparing the clinical characteristics in various risk groups. The R package “limma” (FDR <  0.001) is adopted to recognize the differentially expressed genes (DEGs) between different subtypes.

## 2. Establishment and Verification of a Prognostic Pyroptosis-Associated Gene Signature

The TCGA samples are divided into two groups at 1 : 1 randomly: training cohort and internal validation dataset [13–15]. Genes related to OS in the training cohort are identified with univariate Cox regression exploration, and the filter *p*-value is set as *<*0.05. The least absolute shrinkage and selection operator (LASSO) algorithm are adopted to eliminate the overfitting between the prognosis-associated genes, to decrease the range of the prognosis-associated genes with penalty coefficient tuning conducted *via* 10-fold cross-verification on basis of the R package “glmnet”. The patients at low and high risks are divided into the groups on basis of the average risk mark.  Table 1 shows the clinicopathological features between training and internal verification cohorts.

Personal normalized gene expression values weighted by their LASSO-Cox parameters are included to establish a risk mark model. The calculation of risk mark of every sample is made on the basis of our formula, and the R package of “timeROC” is adopted to plot the risk mark distribution. Next, the samples are put into the groups at high and low risks by the average value of the risk mark. The survival diversity between the two groups is compared with a long-rank test. The Kaplan–Meier (KM) survival curve is adopted to make the OS of every group. The “prcomp” role in the “stats” R package is adopted to make PCA on the basis of the 2-gene signature.

Functional enhancement exploration of the DEGs between the groups was perfomed [16–19]. The samples are put into two subgroups based on the average risk mark. The filtering of DEGs between the groups at low and high risks is made on basis of given standards (|log2FC| ≥ 1 and FDR < 0.05). On the basis of these DEGs, the ssGSEA is made with the “gsva” package to calculate the marks of infiltrating immune cells and to assess the activity of immune-associated paths.

## 3. Experimental Results

### 3.1. Recognition of DEGs in the TCGA Cohort between Normal and Tumor Tissues

The comparison of 52 pyroptosis-associated gene expression extents is made in the TCGA cohort between normal and tumor tissues, and 42 differentially expressed genes (DEGs) (all *p* < 0.05) are recognized.  Figure 1 shows the expressions of the 33 pyroptosis-associated DEGs and the mutual effects among them.

### 3.2. Tumor Classification on the Basis of the DEGs

All HCC patients could be classified into different clusters on basis of 42 DEGs with various clinical coefficients and prognosis.  Figure 2 shows tumor categorization on the basis of the pyroptosis-associated DEGs.

### 3.3. Constructing a Prognostic Risk Model and the HCC Tissue Validation

First, the construction of risk mark model is made on basis of the training cohort. Univariate Cox regression is made on every DEG. There are 154 genes recognized as risk elements for the OS of HCC patients. Next, the number of genes is narrowed with LASSO-Cox regression exploration for constructing our risk mark model. There are two genes in this model. The model formula is given below: Risk mark = 0.406*∗*CEP55 + 0.022*∗*MMP1. According to the abovementioned formula, the high expression extents of *CEP55* and *MMP1* as risk elements of prognosis are related to high risk. The allocation of every patient's risk mark is acquired after calculating the risk mark of every patient in the training cohort. According to the principal component analysis (PCA), patients with various risks are well isolated into two clusters. A positive association between risk mark and death is shown. The analysis of formula's prognosis forecast potency is made for 1, 2, and 3 years according to Figure 3(f). The model showed a relatively high value of region under the curve (AUC): above 0.805. Besides, patients in the training cohort are put into the groups at low and high risks on basis of their risk marks. The KM curves of survival are also made in Figure 3. A great diversity in survival possibility between the two groups (*P* = 0.003) is discovered according to Figure 3. Patients with marks at high risks are related to greatly worse OS, indicating that the high-risk mark is a harmful prognostic element. Figure 3 shows the construction of risk signature in the TCGA training cohort.

### 3.4. Internal and External Verification to Assess the Robustness of the Risk Model

Figure 4 is the internal verification. First, the robustness of the risk model that is constructed above is verified with the TCGA internal validation cohort in Figure (a). The PCA displayed qualified isolation between the two subgroups in Figure (b). Figures 4(a) and 4(c) display that high-risk mark patients showed worse OS which conformed to that of the training cohort. ROC curves displaying the effectiveness of prognosis forecast for 1-, 2-, and 3- years in the three external verification cohorts are shown in Figure 4(e). Moreover, the potency of prognosis forecast for 1, 2, and 3 years in the internal verification cohort is analyzed by generating PRC curves according to Figure 4(e). The model showed a great AUC of above 0743. On basis of the median risk mark, patients are put into the groups at high and low risks. The KM curves are adopted for the comparison of the OS of the two groups in Figure 4(d). The high-risk group patient showed obviously worse survival results by comparing with those from the low-risk group (*p* < 0.001). One external dataset is adopted for assessing the robustness of the risk model applying the ICGC dataset. Similar outcomes that high-risk mark is associated with worse OS are acquired in ICGC cohort. The model showed a relatively high differentiating capacity of prognosis and could recognize the high-risk group patients with worse survival outcomes in ICGC cohort. Two groups show great diversities with the *p* < 0.001 in the ICGC cohort.

### 3.5. Independent Prognostic Value of the Risk Model

Whether the risk mark originated from the gene signature model could be employed as an independent prognostic element is evaluated with univariate and multivariable Cox regression explorations. According to the univariate Cox regression exploration, the risk mark is an independent element forecasting poor survival in among the TCGA training, TCGA internal validation, and ICGC cohorts (HR = 9.886, 95% CI: 4.260–22.943, HR: 5.519, 95% CI: 2.298–13.258 and HR: 5.265, 95% CI: 2.676–10.359). The multivariate exploration also indicated that after modifying for other confounding elements, the risk mark is a prognostic element (HR = 7.657 95% CI: 2.930–20.012, HR = 3.773 95% CI: 1.461–9.740, and HR: 4.508, 95% CI: 2.221–9.150) for patients with HCC in three cohorts. Moreover, after generating a heatmap of clinical characteristics for the TCGA cohort, the diversely distributed degrees of tumor differentiation tumor stage between the subgroups (*p* < 0.05) at low and high risks are observed.  Figure 5 shows external verification.

### 3.6. Immune Status and Tumor Microenvironment Analysis

For exploring the association between the risk mark and immune situation, the enhancement marks of diverse immune cell subpopulations, associated roles, or paths with ssGSEA are quantified. To be interesting, the antigen presentation process, such as the mark of APC_co_stimulation, CCR, MHC_class_I, T_cell_co-stimulation, aDCs, Macrophages, Tfh, Th1_cells, and Th2_cells, are obviously varied between the groups at low and high risks in the TCGA training cohort (all modified *p* < 0.05). Besides, the type II IFN answer and NK cells showed a lower mark in the group at high risks, while the activity of checkpoint molecules, the marks of macrophages, or Treg cells are just the opposite (modified *p* < 0.05). The outcomes of comparisons in the TCGA internal verification cohort are like those in the TCGA training cohort between the two risk groups.  Figure 6 shows the cox regression explorations for the risk mark.  Figure 7 shows the heatmap for the risk groups.  Figure 8 shows the comparing the ssGSEA marks for immune cells and immune paths.

## 4. Data Analysis, Results, and Discussion

Chronic infection of the liver results in the gradual growth of hepatitis and liver cirrhosis, thus boosting the progression of HCC. Because HCC is a greatly heterogeneous primary tumor in the liver, conventional tumor staging approaches cannot forecast HCC prognosis well. Recently, increasing attention has been paid to molecular typing of tumors. A large body of molecular signatures related to HCC have been set up. Hence, the association between the prognosis and mechanisms of GC cells is explored to facilitate treatment.

Hepatocellular carcinoma (HCC) is a common and highly malignant liver tumor with the highest incidence in Asia and Africa where hepatitis virus is prevalent; however, the incidence of liver cancer in North America and Europe has also been increasing in recent years. Although only a small tumor can be completely removed by surgery in some patients, the prognosis is still poor. In recent years, many biological prognostic molecular markers combined with clinical indicators have been discovered. So far, there is no research to compare the predictive ability of these molecular markers. Staging systems based on clinical parameters have been shown to have limited predictive value for prognosis. In order to improve the predictive ability of the clinical staging system, researchers have explored the integration of different predictors into the original model. Currently, more than 10 prognostic staging systems have emerged, including the TNM staging system, the Vauthey simple liver cancer staging system, the Izumi-improved staging system for tumor metastasis, CLIP system staging system, CUPI prognostic index staging system, JIS staging system, BCLC staging system, and French staging system. The Okuda staging system is widely used because of its simplicity and reliability and is still considered to be the most successful staging system. TNM staging has achieved great success in tumor staging other than liver cancer. However, because it mainly considers the factors of the tumor itself, the lack of consideration for the external factors of the tumor (such as liver function reserve, etc.) largely limits its application in liver cancer. Such improved staging systems (e.g., CUPI staging) add clinical features (e.g., ascites) and symptoms to TNM staging. Takanishi et al. compared the existing staging systems and found that CLIP staging has a good performance for prognosis prediction. However, some researchers believe that CLIP staging is not significant for guiding postoperative treatment. Marrero et al compared 7 staging systems through the prognostic follow-up of 239 patients with liver cancer after surgery, found that clinical status, tumor size, liver function, and treatment are independent factors affecting tumor prognosis and found that the BCLC staging system included almost all factors. Cases perform best. In conclusion, different staging systems have their own advantages. The combined application of different prognostic factors and the search for more effective prognostic factors are still the hope of liver cancer prediction.

In this paper, 42 DEGs are screened out from the TCGA. On the basis of the expression level of 42 DEGs, the training cohort, is clustered into two subtypes. For exploring the molecular diversities among various subtypes, the DEGs of the different subtypes are identified further. According to univariate Cox analysis, 154 of DEGs are related to overall survival. LASSO regression exploration is adopted to set up a prognostic model combining 2 pyroptosis-related genes (CEP55 and MMP1). On the basis of the median risk mark, patients are put into the groups at low and high risks. According to the multivariate Cox regression exploration, a risk mark is an independent predicting agent for OS. Immune status is related by further evaluating the risk score. As a midbody-associated protein of 55 kDa, CEP55 (Centrosomal Protein 55) consists of 464 amino acids and exerts a significant effect on controlling the DNA damage and physical cytokinesis. The CEP55 overexpression has been associated with a poor prognosis and has been shown to increase tumor cell motility and invasion for lung cancer, esophageal squamous cell carcinoma, breast cancer cells, and osteosarcoma. Similar outcomes are discovered in liver cancer. Upregulation of CEP55 predicts dismal prognosis in patients with liver cancer. CEP55 drives cell motility via JAK2-STAT3-MMP cascade in hepatocellular carcinoma. Upregulating CEP55 forecasts dismal prognosis among patients with liver cancer. In the current research, there is a CEP55 gene in our risk model.

Under normal circumstances, the positive rate of MMP-1 is very low, but it can be highly expressed under various stimuli. Researches have displayed that great expression of MMP-1 is correlated with prognosis in malignant tumors. Our research illustrated that overexpression of MMP-1 could grow the risk of survival in HCC.

## 5. Conclusion

Two pyroptosis molecular subtypes among HCC patients with various prognosis are observed. A two-gene signature-related risk model with an excellent prognostic forecast is constructed in HCC patients. Our model is made up of two genes, and few genes shall be adopted for prognostic forecast in models. However, our research had some restrictions. First, our outcomes are on the basis of public databases without our own cohort data for validation. Second, our findings lack experiments validations. Finally, our findings shall be confirmed by more preclinical researches and potential clinical tests.

## Figures and Tables

**Figure 1:** Expressions of the 33 pyroptosis-associated DEGs and the mutual effects among them.

**Figure 2:** Tumor categorization on the basis of the pyroptosis-associated DEGs.

**Figure 3:** Construction of risk signature in the TCGA training cohort.

**Figure 4:** Internal verification: (a) Allocation of patients; (b) PCA plot; (c) Survival situation for every patient; (d) Kaplan–Meier curves; and (e) ROC curves.

**Figure 5:** External Verification: (a) Allocation of patients; (b) PCA plot; (c) Survival situation for every patient; (d) Kaplan–Meier curves; (e) Time-dependent ROC curves.

**Figure 6:** Cox regression explorations for the risk mark: (a) Univariate analysis; (b) multivariate analysis; (c) univariate exploration for the TCGA internal verification cohort; (d) multivariate exploration for TCGA Internal verification cohort; (e) univariate exploration for the ICGC verification cohort; and (f) multivariate analysis for ICGC verification cohort.

**Figure 7:** Heatmap for the risk groups.

**Figure 8:** Comparison of the ssGSEA marks for immune cells and immune paths.

**Table 1:** Clinicopathological features between training and internal verification cohorts.

Characteristics		Total	TCGA training cohort	TCGA internal validation cohort	*p*-value
Age	≤65	187 (66.55%)	95 (65.52%)	92 (67.65%)	0.801
	>65	94 (33.45%)	50 (34.48%)	44 (32.35%)	

Gender	Female	83 (29.54%)	40 (27.59%)	43 (31.62%)	0.542
	Male	198 (70.46%)	105 (72.41%)	93 (68.38%)	

Grade	G1-2	181 (64.41%)	87 (60%)	94 (69.12%)	0.137
	G3-4	98 (34.88%)	57 (39.31%)	41 (30.15%)	
	Unknow	2 (0.71%)	1 (0.69%)	1 (0.74%)	

Stage	Stage I-II	202 (71.89%)	104 (71.72%)	98 (72.06%)	0.996
	Stage III-IV	67 (23.84%)	35 (24.14%)	32 (23.53%)	
	Unknow	12 (4.27%)	6 (4.14%)	6 (4.41%)	

T	T1-2	215 (76.51%)	110 (75.86%)	105 (77.21%)	0.998
	T3-4	64 (22.78%)	33 (22.76%)	31 (22.79%)	
	Unknow	2 (0.71%)	2 (1.38%)	0 (0%)	

M	M1	216 (76.87%)	115 (79.31%)	101 (74.26%)	0.995
	M0	1 (0.36%)	1 (0.69%)	0 (0%)	
	Unknow	64 (22.78%)	29 (20%)	35 (25.74%)	

N	N0	198 (70.46%)	106 (73.1%)	92 (67.65%)	1
	N1	4 (1.42%)	2 (1.38%)	2 (1.47%)	
	Unknow	79 (28.11%)	37 (25.52%)	42 (30.88%)	

## Data Availability

The simulation experiment data used to support the findings of this study are available from the corresponding author upon request.
